The article "The effect of n-3/n-6 polyunsaturated fatty acids on acute reflux esophagitis in rats" was retracted in 2023. Reasons: duplicated images; original data or images not available; unreliable data; unreliable results or conclusions.

# The effect of n-3/n-6 polyunsaturated fatty acids on acute reflux esophagitis in rats

**DOI:** 10.1186/s12944-016-0332-2

**Published:** 2016-10-04

**Authors:** Ze-Hao Zhuang, Jing-Jing Xie, Jing-Jing Wei, Du-Peng Tang, Li-Yong Yang

**Affiliations:** 1 Department of Endoscopy, The First Affiliated Hospital of Fujian Medical University, 20 Chazhong Road, Fuzhou, 35005 China; 2 Department of Endocrinology, The First Affiliated Hospital of Fujian Medical University, Fuzhou, 35005 China

**Keywords:** Acute reflux esophagitis, Rat model, n-3/n-6 polyunsaturated fatty acids, Lipid peroxidation

## Abstract

**Background:**

Polyunsaturated fatty acids (PUFAs) play various roles in inflammation. However, the effect of PUFAs in the development of reflux esophagitis (RE) is unclear. This study is to investigate the potential effect of n-3/n-6 PUFAs on acute RE in rats along with the underlying protective mechanisms.

**Methods:**

Forty Sprague Dawley rats were randomly divided into four groups (*n* = 10 in each group). RE model was established by pyloric clip and section ligation. Fish oil- and soybean oil-based fatty emulsion (n-3 and n-6 groups), or normal saline (control and sham operation groups) was injected intraperitoneally 2 h prior to surgery and 24 h postoperatively (2 mL/kg, respectively). The expressions of interleukin (IL)-1β, IL-8, IL-6 and myeloid differentiation primary response gene 88 (MyD88) in esophageal tissues were evaluated by Western blot and immunohistochemistry after 72 h. The malondialdehyde (MDA) and superoxide dismutase (SOD) expression in the esophageal tissues were determined to assess the oxidative stress.

**Results:**

The mildest macroscopic/microscopic esophagitis was found in the n-3 group (*P* < 0.05). The expression of IL-1β, IL-8, IL-6 and MyD88 were increased in all RE groups, while the lowest and highest expression were found in n-3 and n-6 group, respectively (*P* < 0.05). The MDA levels were increased in all groups (*P* < 0.05), in an ascending trend from n-3, n-6 groups to control group. The lowest and highest SOD levels were found in the control and n-3 group, respectively (*P* < 0.05).

**Conclusion:**

n-3 PUFAs may reduce acute RE in rats, which may be due to inhibition of the MyD88-NF-kB pathway and limit oxidative damage.

## Background

Gastro-esophageal reflux disease (GERD) is a chronic disease involving mucosal damage and epithelial metaplasia, which is caused by gastric and duodenal contents entering the esophagus. Reflux esophagitis (RE) is one of the important clinical sub-types of GERD [1]. Several animal models of RE have been established successfully, including Pyloric Nylon Loop-induced Chronic Acid Reflux Esophagitis (PNL-CARE) model, which uses a modified protocol based on our previously published Pyloric Clip-induced Chronic Acid Reflux Esophagitis (PC-CARE) model [2].

It was traditionally believed that the onset of RE was caused by directly chemical injury on mucosa [3]. However, studies have demonstrated that inflammatory factors, such as interlukin-6 (IL-6), interlukin-8 (IL-8), and interlukin-1β (IL-1β) are also elevated in patients with non-erosive reflux disease (NERD), which has no macroscopic esophageal mucosal damage [4, 5]. These observations suggest that inflammatory cytokines and the resulting oxidative stress may play an important role in the development of RE.

Oxyradicals generated by esophageal acute inflammatory cells and vascular endothelial cells, including lipid peroxidation (LPO)-induced oxidative stress, are involved in the development of acute RE in GERD patients [6]. This suggests that modulating LPO may be an effective way to control the development of RE [7, 8].

Polyunsaturated fatty acids (PUFAs) are divided into several subclasses, including n-3 or n-6 according to the location of the double bond. These PUFAs play various roles in the development of inflammation. Studies have shown that n-3 PUFAs inhibit the expression of toll-like receptors (TLRs) in order to downregulate myeloid differentiation primary response gene 88 (MyD88)-nuclear factor - kappa B (NF-kB) signal transduction, and decrease the levels of pro-inflammatory factors, such as tumor necrosis factor-α (TNF-α), IL-β, IL-6 and IL-8 in acute RE [9–11]. Studies conducted on mice and humans suggest that diets supplemented with n-3 PUFAs have significant anti-oxidative effects, while linseed oil (abundant in n-3 PUFAs) also showed significant anti-oxidative and anti-ulcer effects [12]. However, n-6 PUFA is believed to be a pro-inflammatory substance.

In this study, we observed the effect of intraperitoneally administered n-3 or n-6 PUFA on the expression of inflammatory factors and LPO indices, along with the underlying protective mechanisms, in rats with acute RE.

## Methods

### Reagents

Ten percent soybean oil-based lipid emulsion (Intralipid Injection) and 10 % n-3 fish oil-based lipid emulsion (Omegaven Injection) were purchased from Sino-Swed Pharmaceutical Corp. Ltd., Wuxi, China. Superoxide dismutase (SOD) and malondialdehyde (MDA) assays were purchased from Nanjing Bioengineering Co. Ltd., Nanjing, China. The antibodies of IL-1β, IL-8, IL-6 and MyD88 were purchased from Abcam. Plc, Shanghai, China. Triglyceride (TG) and total cholesterol (TC) assays were bought from Eastern Diagnostic Products Co. Ltd, Anji, China. Reagents of immunohistochemistry and diaminobenzidine tetrahydrochloride (DAB) assay to detect IL-1β, IL-8 and MyD88 expression were bought from Zhongshan Golden Bridge Biotech. Ltd. Co, Beijing, China.

### Establishment of rat models

Male Sprague Dawley (SD) rats (6–8 weeks old), weighing 240 ± 10 g, were procured from the Laboratory Animal Center of Fujian Medical University. The experimental procedures, and the animal use and care protocols were approved by the Committee on Ethical Use of Animals of The First Affiliated Hospital of Fujian Medical University. Briefly, under chloral hydrate by intraperitoneal injectionanesthesia using chloral hydrate by intraperitoneal injection in about 40 rats that underwent overnight fasting, the RE model was established by a modified protocol based on PC-CARE model [2]. In brief, the edge of the forestomach and glandular stomach of rat was ligated by 3-0 non-absorbable suture (Johnson Medical Ltd. Shanghai, China) and the pyloric ring were occluded by pyloric clip to achieve incomplete obstruction of the pylorus (the diameter of the pyloric ring after occlusion was 4.2 mm). In the sham operation group, the stomach and duodenum were dissociated for 2 min without ligating the pylorus and duodenum.

Forty SD rats were randomly divided into four groups, including sham operation group, control group, n-3 PUFAs group and n-6 PUFAs group, with 10 rats in each group. Two mL/kg 0.9 % normal saline (NS) was injected intraperitoneally to the sham operation group and control group. The n-3 and n-6 PUFAs groups were injected intraperitoneally with 2 mL/kg fish oil-based lipid emulsion and 2 mL/kg soybean oil-based lipid emulsion, respectively. These injections were given totally for four times: 2 h before surgery, and 22, 46 and 70 h after surgery. Any death occurring after surgery was noted. Rats were killed with an overdose of chloral hydrate72 h after surgery.

### Specimen collection

Rats were anaesthetized and blood was collected from inferior vena cava immediately after they were killed. The TC and TG levels were measured by assays within 2 h of drawing of blood. Rats were killed 72 h after the procedure, and esophageal and liver tissues were collected. The esophagus was dissected and 0.9 % NS was used to remove blood by washing repeatedly. The damage of esophageal mucosa was scored from 0 to III according to Kuwahata’s criteria [13]. The grading system was as following: grade 0, normal -appearing esophageal mucosa; grade I, mucosa with erythema; grade II, mucosa with erosion or sloughing; and grade III, mucosa with a thickly coated ulcer, hemorrhage, and/or stricture.

Part of the esophagus was packed by tinfoil and frozen using liquid nitrogen and stored at −80 °C. They were used to assess the protein expression, contents of MDA and activity of SOD.

### Hematoxylin and eosin staining

Esophageal and liver tissues were fixed for 24 h in 10 % neutral formalin and after dehydration, were embedded in paraffin and sliced, stained with hematoxylin and eosin (H&E) and observed under an optical microscope (100× and 400×). HE staining of esophageal inflammation were scored from – to +++, in the following manner: -, no inflammatory cells infiltration; +, less than 5 cells per field mild lesions; ++, 5~10 cells per field; +++, more than 10 cells per field.

### IL-1β, IL-8 and MyD88 protein detection

The concentration of proteins extracted from the tissues was measured by bicinchoninic acid assay (BCA) and detected by Western blot. In brief, the esophageal tissue (100 mg) was obtained and added to 1.0 ml of cell lysis buffer [20 mM Tris–HCl (pH 7.4), 150 mM NaCl, 1 mM EDTA, 1 mM EGTA, 1 % Triton X-100, 2.5 mM sodium pyrophosphate, 1 mM ß-glycerophosphate, 1 mM Na_3_VO_4_, 1 μg/ml leupeptin, 1 μg/ml aprotinin, 1 μM PMSF], and protein concentrations were measured using D_C_ Protein Assay kit (Bio-Rad, Hercules, CA). Equal amount of protein (30 μg) was loaded onto a SDS–polyacrylamide gel for electrophoresis and then transferred on a PVDF membrane (Amersham, Piscataway, NJ). The blots were immersed in 5.0 % milk (prepared with milk powder) for 1 h. Then at 4 °C rabbit anti-IL-1β, IL-8 and MyD88 antibodies at dilutions of 1:300 or β-actin at dilutions of 1:1000 were added to the blots, which were then incubated overnight. After washing with TBS-T, the membrane was incubated with secondary antibodies and the signals were visualized by ECL system (Amersham). The relative amounts of each protein were quantified by densitometry as ratios to b-actin.

### IL-1β, IL-8 and IL-6 expression detected by immunohistochemistry

IL-1β, IL-8 and IL-6 expression were detected by immunohistochemistry and DAB assay. The procedures were performed according to the reagent manufacturer’s instructions. In brief, after antigen retrieval, endogenous peroxidase activity was blocked with 3 % hydrogen peroxide for 15 min at 37 °C. After being restored, blocking agent (10 % normal goat serum) was added to dissolve the slices at room temperature. Thirty minutes later, rabbit anti-IL-1β, IL-8 and IL-6 were added at a dilution of 1:100 at 4 °C. The slices were then incubated overnight and washed thrice with phosphate buffered saline (PBS) for 10 min each, the next day. At room temperature, general secondary antibody was added, and the slices were incubated at 37 °C for 30 min. After washing, streptavidin-peroxidase was added at 37 °C. Thirty minutes later, the slices were then stained with 3,3-diaminobenzidine for 5 min. Sections were counterstained with haematoxylin. These slices of mucosa of RE were observed under the microscope for the measurement of expression of IL-1β, IL-8 and IL-6.

### Levels of MDA and the activity of SOD detection

Esophageal tissue homogenate was used for the detection of MDA level and the activity of SOD. The detection followed the manufacturer’s instructions.

### Levels of TC and TG detection

Serum was used for the detection of TC and TG levels. The detection followed the manufacturer’s instructions.

### Results determination

On immunohistochemical analysis, the expression of IL-1β, IL-8 and IL-6 were mainly located in the cytoplasm and mesenchyma. The criterion of IL-6 expression was according to the method described by Nakano et al. [14]. No positive cells was considered as negative; positive cells <25 % was considered as weakly positive; positive cells between 25 and 75 % was considered as medium positive and positive cells >75 % was considered as strongly positive.

### Statistical analysis

SPSS 19.0 software was used for analysis of data. Quantitative data were represented as mean ± standard deviation. Intra-group significance was compared using student’s *t*-test. Multi-group comparison was done using one-way ANOVA and multiple comparisons among the groups were done by least-significant difference (LSD). Categorical data was represented by constituent ratio and analyzed by *χ* ^2^ test. Correlation analysis was represented by Pearson correlation analysis. Ranked data was analyzed by rank sum test and inspection level was 0.05. Results were considered statistically significant when *P* < 0.05.

## Results

### Basic conditions of the rats

Four of the 40 rats were found dead, including one from severe aspiration pneumonia and 3 of esophageal perforation, which leads to pulmonary abscess. There was no significant difference in the survival ratio after surgery among the 4 groups (*P* = 0.539).

### The degree of esophagitis among groups

The esophageal mucosa of rat was smooth and without macroscopic lesions in the sham operation group. The stomachs of the rats in all the three modeled groups were full and expanded and the esophagus had erosion of varying degrees. The most serious manifestation of erosive esophagitis presented with a large ulcer, necrosis and bleeding. Majority of the lesions were located in the middle and lower sections of the esophagus. Histological examination of esophageal mucosa was normal in the sham operation group. However, on histological examination of esophagus from all the three RE groups, epithelial defects and inflammatory cell infiltration were seen under the microscope. Several neutrophils, eosinophils, and monocytes were seen under high magnification (Fig. 1).

**Fig. 1:** Gross specimen (**a**) and hematoxylin and eosin (H&E) staining of esophageal mucosa (**b**) 72 h after surgery in sham operation group (*left*) and RE model groups (*right*); normal esophageal epithelial and a small quantity of inflammatory cells were seen in sham operation group; Lower ulcer with peripheral congestion and swelling was seen in RE model groups 72 h after surgery. H&E staining showed that epithelial defects and inflammatory cells infiltration. Several neutrophils, eosinophils, and monocytes were seen under high magnification

### Macroscopic grading of changes in rat esophagus

The morphological grading in different groups were significantly different when analyzed using rank-sum test (*P* = 0.031). Ranked data were compared using LSD test and significant difference was found between n-3 and n-6 PUFA groups (*P* = 0.008) and no significant difference was found in the other groups (*P* > 0.05, Table 1, Fig. 2).

**Table 1:** Grade of damage to esophageal mucosa

Group	Grade (*n*/*n*%)			
	0	I	II	III
n-3 PUFAs	4/44.4 %	2/22.2 %	0	3/33.3 %
n-6 PUFAs	0	1/12.5 %	0	7/87.5 %
Control	0	1/11.1 %	3/33.3 %	5/66.7 %
Sham operation	10	0	0	0

*PUFA* polyunsaturated fatty acids

**Fig. 2:** Macroscopic observation of the degree of esophagitis. **a** Sham operation group; **b** n-3 PUFA group; **c** Control group; **d** n-6 PUFA group. The esophageal mucosa is smooth in sham operation group, while bleeding and perforation occurred in n-6 PUFA groups. The degree of mucosa damage increased from **a** to **d**

### Histological grading of esophageal changes in different groups

The grading of H&E staining among the groups showed significant difference when analyzed by rank-sum test (*P* = 0.027). Ranked data was compared using LSD test and significant difference was found between n-3 PUFA and n-6 PUFA (*P* = 0.007), n-3 PUFA and control group (*P* = 0.042). There were no significant differences among other groups (*P* > 0.05, Table 2, Fig. 3).

**Table 2:** Grade of H&E staining of inflammation

Group	Grade (*n*/*n*%)			
	−	+	++	+++
n-3 PUFAs	3/33.3 %	3/33.3 %	1/11.1 %	2/22.2 %
n-6 PUFAs	0	1/12.5 %	1/12.5 %	6/75.0 %
Control	0	1/11.1 %	4/44.4 %	4/44.4 %
Sham operation	10	0	0	0

**Fig. 3:** H&E staining of esophagitis under microscopy. **a** Normal esophageal epithelial with stratified squamous epithelium (H&E staining, 100×); **b** Inflammatory cells were seen under high magnification (H&E staining, 100×); **c** Epithelial defects in acute RE models. **d** Numerous neutrophilic granulocytes, eosinophilic granulocytes, and monocytes were seen under high magnification (H&E staining, 400×). **e** Some mucosal disruptions occurred including ulcer, necrosis, and bleeding (H&E staining, 400×). The *arrow* represents neutrophils

### Expression of IL-1β, IL-8 and MyD88 in different groups by Western blot

The levels of IL-1β, IL-8 and MyD88 in all the 4 groups were measured using western blot analysis. Compared with the sham operation group, the expression levels of IL-1β, IL-8 and MyD88 were significantly higher in all the three RE model groups (*P* < 0.01). The expressions were lowest in n-3 PUFAs group and highest in n-6 PUFAs group and statistically significant differences were found when compared with other groups (*P* < 0.05, Fig. 4). Pearson correlation analysis showed that MyD88 was significantly correlated with both IL-1β (*P* < 0.05, *r* = 0.844) and IL-8 (*P* < 0.05, *r* = 0.684).

**Fig. 4:** **a** The protein expressions of IL-1β, IL-8 and MyD88 in respective groups; **b** The protein expressions of IL-1β, IL-8 and MyD88 were significantly higher in model groups; their expressions were lowest in n-3 PUFAs group and highest in n-6 PUFAs group; (*: *P* < 0.05 vs sham operation group;# : *P* < 0.05 vs other model groups)

### Immunohistochemistry of IL-1β, IL-8, and IL-6 in different groups

The expressions of IL-1β and IL-8 were negative in normal esophageal epithelium but positive in esophagitis tissues. The positive-staining was located in the cytoplasm of squamous cells and submucosal inflammatory cells, lamina propria and region of inflammatory infiltration.

The expression of IL-6 was negative in normal esophageal epithelium and those with esophagitis, but positive in sub-epithelial structures in esophagitis. The positive-staining was located in the cytoplasm of submucosal inflammatory cells, lamina propria and regions of inflammatory infiltration.

The protein level of IL-6 as examined by immunohistochemistry in the esophagus was significantly higher in all three RE model groups when compared with sham operation group (*P* < 0.05). IL-6 expression was lowest in n-3 PUFAs group and highest in n-6 PUFAs group (*P* < 0.05, Table 3, Fig. 5).

**Table 3:** The expression of IL-6 protein by immunohistochemistry

Group	Grade (*n*/*n*%)			
	−	+	++	+++
n-3 PUFAs	4/44.4 %	3/33.3 %	2/22.2 %	0
n-6 PUFAs	0	2/25.0 %	4/50.0 %	2/25.0 %
Control	1/11.1 %	5/55.6 %	2/22.2 %	1/11.1 %
Sham operation	10	0	0	0

*PUFAs* polyunsaturated fatty acids

**Fig. 5:** IL-1β, IL-8 and IL-6 expression were examined by immunohistochemistry in different groups. IL-1β (**a**), IL-8 (**b**) and IL-6 (**c**) expressions were negative in sham operation group; IL-1β (**d**), IL-8 (**e**) and IL-6 (**f**) expressions were positive in acute RE groups, which were stained in sepia

### Level of MDA and the activity of SOD in different groups

The level of MDA expression, a marker of lipid peroxidation during oxidative stress was significantly higher in all three RE model groups when compared with the sham operation group (*P* < 0.01). Its level was lowest in the n-3 PUFAs group and highest in the control group and a significant difference was found when compared with other groups (*P* < 0.05). The activity of SOD, an enzyme crucial for preventing damage due to oxidative stress, was significantly lower in the control group when compared with the sham operation group (*P* = 0.022). Higher activity of SOD was found in the n-3 PUFA group when compared to the other groups (*P* < 0.05, Table 4).

**Table 4:** SOD and MDA expressions in esophageal tissue

Group	MDA (nmol/mg prot)	SOD (U/mg prot)
n-3 PUFAs	1.3 ± 0.36*#	41.6 ± 2.67*#
n-6 PUFAs	2.1 ± 0.26*Δ	32.3 ± 7.69
Control	2.5 ± 0.54*	28.5 ± 6.05*
Sham operation	0.7 ± 0.42	35.2 ± 7.24

*P < 0.05 *vs* sham operation group; #*P* < 0.05 *vs* other groups; Δ*P* < 0.05 *vs* control groups; *MDA* malonaldehyde, *SOD* superoxide dismutase, *PUFA* polyunsaturated fatty acids

### Levels of TG and TC in different groups

The serum levels of TC and TG in different groups were compared by one-way ANOVA, while the LSD was used for the comparison among groups. TG levels were significantly decreased in the n-3 PUFA group, compared with the sham operation group (*P* = 0.039) and control group (*P* = 0.001). Other groups had no significant differences in TG levels (*P* > 0.05). TC levels were significantly lower in the n-3 PUFAs group compared with other groups (*P* < 0.005), while no significant differences were found in other groups (*P* > 0.05, Table 5).

**Table 5:** TC and TG concentration in plasma

Group	TG (mmol/l)	TC (mmol/l)
n-3 PUFAs	1.37 ± 0.4*Δ	1.38 ± 0.18▲
n-6 PUFAs	1.71 ± 0.58	1.94 ± 0.33
Control	2.13 ± 0.28	1.76 ± 0.19
Sham operation	1.84 ± 0.59	1.73 ± 0.2

*P < 0.05 *vs* sham operation group; Δ*P* < 0.05 *vs* control group; ▲*P* < 0.05 *vs* other groups; *TG* triglycerides, *TC* total cholesterol, *PUFA* polyunsaturated fatty acids

### H&E staining of liver tissues in different groups

Only one rat in n-6 PUFAs group had fatty infiltration of liver tissue and no other rats had fatty infiltration of liver tissues (Fig. 6).

**Fig. 6:** **a** H&E staining in normal liver (×400); **b** HE staining in fatty liver (×400), and there was adipose degeneration in liver cells with bright round lipid droplet. The *arrow* represents liver cells with adipose degeneration

## Discussion

In the present study, we established a modified protocol based on PC-CARE^2^ model in SD rats to induce acute RE. Macroscopic changes consistent with RE were found in all the modeled rats 72 h after surgery in control group, which were confirmed by histological examination. The survival rate was over 80 % at 72 h after surgery, which suggests the method used in this study was reliable, with a low mortality rate. Further, this procedure is simple to perform and has minimal adverse effects on the gastrointestinal function.

In this experiment, the morphological grading of the esophagus and histological grading H&E stained esophageal sections showed that esophageal damage and inflammation were markedly decreased in the n-3 PUFA group (*P* < 0.05), while the proportion of grade III damage in n-6 PUFAs group was significantly higher than other RE model groups (7/8, 87.5 %), which suggested that n-3 PUFA reduced inflammation and reflux-related damage, while n-6 PUFA increased inflammation. Although the exact time of acute RE could not be estimated, the acute inflammation in esophageal mucosa during GERD is persistent and is the initial step before development of chronicity [15]. Consequently, n-3 PUFA may be a potential treatment option to prevent and control GERD.

Besides direct damage caused by gastroesophageal reflux, there are many neutrophils located in the mucosal and submucosal layers which could generate reactive oxygen species (ROS) and induce oxidative stress and cytokine-mediated damage [16]. As an early inflammatory factor, IL-8 could be stimulated by reflux and the expression of which is significantly associated with the severity of RE [17, 18]. IL-1β expression is another important cytokine which is related to RE and its expression is significantly higher in RE models compared with controls [19]. IL-6, as an acute phase reactant, is induced by mononuclear phagocytes, vascular endothelial cells and fibroblasts, upon stimulation by IL-1β and TNF-α. Studies showed that esophageal cell suspension had significantly elevated IL-6 in vitro from RE patients [20].

The present study showed that the protein expressions of IL-1β, IL-8 and IL-6 in RE model groups were significantly higher (*P* < 0.05), when compared to the sham operation group. However, the lowest and the highest expressions were found in n-3 and n-6 PUFAs group, respectively (*P* < 0.05), which was in accordance with the grade of esophageal damage. The immunohistochemical results suggested that IL-8 and IL-1β were extensively expressed in esophageal squamous epithelium, lamina propria and regions of inflammatory cell infiltration in submucosa when acute esophagitis occurred, which suggested that IL-8 and IL-1β play important roles in acute RE. In a study by Yamaguchi et al. [21], it was observed that the IL-6 secretion of esophageal epithelial cells in rats was stimulated by gastroesophageal reflux. However, in our study, IL-6 was only expressed in the lamina propria and regions of inflammatory cell infiltration in the submucosa, but was absent in esophageal squamous epithelium, which suggested that it is not a direct cause for epithelial damage. However, IL-6 expression in submucosa was also observed in some cases without obvious epithelial damages, which suggested that its overexpression along with the up-regulation of IL-8 and IL-1β were early events in acute RE. In contrast to the traditional theory of direct erosion, a large number of cytokines were up-regulated before epithelial damage, suggesting that RE onset may be due to IL-8 and IL-1β stimulated by reflux. Moreover, IL-8 and IL-1β consequently results in esophageal damage and RE progression. Based on this premise, it may be possible to ameliorate the manifestations of RE by inhibiting the inflammatory cascade. We found that administration of n-3 PUFAs could significantly reduce the expressions of IL-1β, IL-8 and IL-6 in acute esophagitis while n-6 PUFAs had opposite effects.

The activation of signal transduction by TLRs and the expression of target gene play a key role in inflammation. A few studies suggested that n-3 PUFAs have anti-inflammatory effects [22, 23]. TLRs combine with pathogen-related molecules non-specifically and activate NF-kB, thus leading to the expression of TNF-α, IL-1β, IL-6, IL-8 and cyclooxygenase-2 (COX-2). During signal transduction through TLR, MyD88 plays a critical role. MyD88 is an important adapter in TLRs signaling pathway and after recognition of the respective ligand by TLRs, MyD88 interacts with the homeodomain and causes activation of the signal cascade. There have been studies regarding roles of TLRs in RE. A few studies suggest that lipopolysaccharides (LPS) of gram negative bacteria dominant in the distal esophagus could be recognized by TLRs, causing a significant increase of NF-kB through MyD88 and the increased cytokines to mucosa damage. The in vitro analysis suggested that TLR3 signaling transduction could increase sensitivity of cells to endogenous signals and thus induce RE [24, 25]. n-3 PUFAs inhibited NF-kB signal transduction through inhibition of MyD88 expression [26]. In vitro analysis showed that n-3 PUFAs could activate NF-kB, which was irritated by TLRs agonist, and inhibit COX-2 expression [27], further down-regulating the expressions of IL-6 and IL-1β [23].

In our study, the expression of MyD88 was significantly higher in all three RE model groups (*P* < 0.05) and its expression significantly correlated with that of IL-1β and IL-8, indicating that MyD88 signaling played an important role in acute esophageal damage. MyD88 activated NF-kB dependent signaling pathway and increased expression of cytokines such as TNF-α, IL-6, IL-1 and IL-8 [28, 29]. MyD88, IL-6, IL-1β and IL-8 were expressed the lowest in the n-3 PUFAs group and highest in the n-6 PUFAs group, suggesting that n-3 PUFAs could significantly decrease MyD88 protein and down-regulate IL-6, IL-1β and IL-8 expression due to inflammation and necrosis inhibition. n-3 PUFA could also protect TLRs activated NF-kB-dependent signaling pathway. Recent studies showed that esophageal bacteria could induce TLRs signaling activation and it is associated with RE and Barrett’s esophagus [30], which provided a new perspective of n-3 PUFAs regulating esophagitis and the relationship with TLRs signaling. However, the present study did not study the effect of bacteria on the RE. Due to the species difference, it is unclear whether the role of the esophageal bacteria to RE is also applicable to humans.

PUFAs are important substrates of oxidative stress [31, 32], while the role of oxidative stress on esophageal epithelial cells in RE has been clearly demonstrated in studies [33]. In the present study, the MDA expression is significantly higher in all model groups (*P* < 0.05), which further supports the role of oxidative stress in acute RE. After reflux irritation, ROS could form LPO through lipid peroxidation by binding with lateral chain of PUFAs or nucleic acids and damaged esophageal mucosa. Free radicals are common links between many signaling pathways [34]. For example, ROS could induce the expression of IL-6, IL-1β and IL-8 by activating NF-kB signaling and damage the esophageal mucosa [35].

The extent of oxidation of fatty acid relies directly on the degree of unsaturation of the double bond. Theoretically, n-3 PUFAs contain more unsaturated ethylenic bond and are more easily oxidized. However, MDA expressed significantly lower in either n-3 or n-6 PUFA treated rats, indicating that PUFA could inhibit lipid peroxidation of esophageal epithelial in acute RE. Similar findings have also been reported in other acute RE models [36]. n-3/n-6 PUFA contain number of ethylene linkages and could provide themselves to free radicals as electron donor and thus, cut off free radical chain reaction. The numbers of double bonds is higher in n-3 PUFAs than that in n-6 PUFAs; therefore, the ability of scavenging free radicals is stronger in n-3 PUFAs than in n-6 PUFAs [37]. In our study, although n-3 and n-6 PUFAs reduced the MDA levels, these levels were lower in the n-3 PUFAs group. On the contrary, the SOD level was significantly higher after n-3 PUFAs treatment, but not n-6 PUFAs, which suggested that n-3 PUFAs remove free radicals by up-regulating antioxidant mechanisms. Additionally, n-3 PUFAs could inhibit pro-inflammatory factors induced by ROS and consequently inhibit acute RE. However, as previously reported, n-6 PUFAs could aggravate acute RE mainly because n-6 PUFAs could slightly decrease the MDA levels and not increase SOD expression, which in turn did not reverse the damage by n-6 PUFAs in acute esophageal damage and cytokines expression.

In the present study, PUFAs were administrated peritoneally and results showed that parenteral lipid emulsion could induce changes in lipometabolism and, thus, lead to increased blood lipid and dysregulated liver function. However, we found that the levels of TC and TG were significantly lower in n-3 PUFAs group compared with controls or other acute RE models (*P* < 0.05), which suggested that n-3 PUFAs had an effect on lowering TG and TC levels. No fatty infiltration in the liver was observed.

The commercial soybean oil-based or fish oil-based lipid emulsion used in this study may represent a potential limit of our study. The commercial emulsions have complex compositions, especially vitamin E, which is added to prevent the production of ROS when fat undergoes oxidation. Though this may raise concerns about the potential influence of the antioxidant function of vitamin E, the concentration of vitamin E in this study was 0.3–0.6 mg/kg, which is far less than the effective antioxidant concentrations in parenteral nutrition studies (50 mg/kg) [38] and is likely to have hardly impact on the ROS of rats.

## Conclusion

Our study suggested that the expressions of IL-6, IL-1β, and IL-8 were increased in acute RE. Additionally, lipid peroxidation was also enhanced. Parenteral administration of n-3 PUFA inhibited acute RE onset without fatty infiltration in the liver. Further, it inhibited MyD88-NF-kB signaling pathway and down-regulate the pro-inflammatory factors. n-3 PUFAs were also found to limit oxidative damage in acute RE by causing a decrease in MDA expression and increase in SOD expression. More studies are required to confirm these findings. The doses at which its benefits can be observed also have to be studied further, in preclinical models as well as in humans.

## Abbreviations

GERD: Gastro-esophageal reflux disease
LPO: Lipid peroxidation
PUFAs: Polyunsaturated fatty acids
TLRs: Toll-like receptors
